The article "Deep Learning Application for Effective Classification of Different Types of Psoriasis" was published in 2022. Journal: J Healthc Eng.

# Deep Learning Application for Effective Classification of Different Types of Psoriasis

**DOI:** 10.1155/2022/7541583

**Published:** 2022-01-15

**Authors:** Syeda Fatima Aijaz, Saad Jawaid Khan, Fahad Azim, Choudhary Sobhan Shakeel, Umer Hassan

**Affiliations:** Department of Biomedical Engineering, Ziauddin University, Faculty of Engineering, Science, Technology and Management (ZUFESTM), Karachi, Pakistan

## Abstract

Psoriasis is a chronic inflammatory skin disorder mediated by the immune response that affects a large number of people. According to latest worldwide statistics, 125 million individuals are suffering from psoriasis. Deep learning techniques have demonstrated success in the prediction of skin diseases and can also lead to the classification of different types of psoriasis. Hence, we propose a deep learning-based application for effective classification of five types of psoriasis namely, plaque, guttate, inverse, pustular, and erythrodermic as well as the prediction of normal skin. We used 172 images of normal skin from the BFL NTU dataset and 301 images of psoriasis from the Dermnet dataset. The input sample images underwent image preprocessing including data augmentation, enhancement, and segmentation which was followed by color, texture, and shape feature extraction. Two deep learning algorithms of convolutional neural network (CNN) and long short-term memory (LSTM) were applied with the classification models being trained with 80% of the images. The reported accuracies of CNN and LSTM are 84.2% and 72.3%, respectively. A paired sample *T*-test exhibited significant differences between the accuracies generated by the two deep learning algorithms with a *p* < 0.001. The accuracies reported from this study demonstrate potential of this deep learning application to be applied to other areas of dermatology for better prediction.

## 1. Introduction

The skin is important for regulating the body's temperature and protects against fungal infection, germs, allergies, and viruses [1]. However, many individuals suffer from skin disorders that stem from various causes. The most common skin disorders include eczema, alopecia, ringworm, and psoriasis [2]. Itchy scaly patches which are red in color and most commonly occur on knees and elbows represent the symptoms of psoriasis. Psoriasis is a persistent skin disorder that cannot be passed from one person to another and has no treatment [3]. According to the International Federation of Psoriasis Associations (IFPA), psoriasis affects 125 million people globally, or around 2% to 3% of the global population [3]. It starts when the autoimmune system of the body begins to attack skin cells, disrupting their regular life and development cycle. Normally, a skin cell develops over a period of 28 to 30 days;, however, in case of psoriasis, this cycle is disturbed and accelerated leading to development of skin cells on the skin surface in 7 days [4]. These excess skin cells develop dense, itchy, swollen, red spots in psoriasis lesions which ultimately spread to several parts of the body. The size of these lesions might range from tiny areas to the full body. The most prevalent forms of psoriasis are pustular, guttate, inverse, plaque, and erythrodermic psoriasis [5]. These tend to exert a substantial detrimental influence on a person's quality of life and are often compared to a heart ailment because they induce depression and are thought to increase the suicide rate by 30% [6]. Dermatologists usually use general observation and biopsies for diagnosis of the correct type of psoriasis. However, the ambiguity surrounding the number of tests required for satisfactory diagnosis regarding the adequate type of psoriasis represent the limitations of the available diagnostic procedures. Hence, there exist immense opportunities for researching new methods in relation to classification and diagnosis of the five types of psoriasis, including pustular, guttate, inverse, plaque, and erythrodermic [7].

Machine learning and deep learning approaches have demonstrated success in the prediction and categorization of a wide range of illnesses. Deep learning involves the use of several computer techniques and reflects the ability to learn and adapt. For diagnostic purposes, machine learning and deep learning technologies have been used in a variety of medical fields. They have shown accuracy in the diagnosis of brain tumors, alopecia areata, Alzheimer's illness, breast cancer, blinding diseases, and renal disease [8–13].

Various deep learning approaches have been used in dermatology to predict and classify skin problems with high accuracy. For categorizing skin images for the identification of skin lesions, such as malignant melanoma, basal cell carcinoma, actinic keratosis, squamous cell carcinoma, and psoriasis, skin analysis algorithms have been developed employing Mask RCNN, transfer learning, and CNN frameworks [14–20]. All of these methods entail the classification of a single kind of skin condition. Furthermore, to the best of our knowledge, none of the deep learning algorithms have been used to classify the five kinds of psoriasis: pustular, guttate, inverse, plaque, and erythrodermic psoriasis.

Hence, in this paper, we propose a deep learning technique for the classification of different types of psoriasis as previous methods have not carried out classification of different types of psoriasis and have used a single deep learning technique. Moreover, previous state-of-the-art works have used different datasets as compared to the datasets that we have used, and we have achieved higher accuracies. Our research motivation and proposal exhibit the practical application of deep learning approaches for distinguishing and classification of five different types of psoriasis including pustular, guttate, inverse, plaque, and erythrodermic. The results from our study also demonstrate the future potential of this deep learning application to be applied to further skin disorders and make dermatological diagnosis more accurate.

## 2. Related Works

Researches have used deep learning approaches for predicting and classifying skin lesions including melanoma and psoriasis. A smart home system was proposed coupled with sensors and artificial intelligence for evaluating skin disorders. The system used normal and melanocytic skin lesion images and applied CNN to achieve an accuracy of 82.4% [15]. In another study, extraction and identification of skin melanoma from dermoscopy images was proposed with the help of VGG-SegNet scheme. The technique used CNN, and the results exhibited an accuracy of 97.16% [16]. In a similar study, skin lesion, in particular, malignant melanoma recognition method was introduced using mask region-based convolutional neural network (RCNN) and transfer learning-based approach. Three datasets including ISBI2016, ISB12017, and HAM1000 were used for validation and presented accuracies of 96.3%, 94.8%, and 88.5%, respectively [14].

Other systems have used multiclass classification along with moth flame optimization for skin lesion segmentation. A system was developed with a fully automated approach with a CNN model. Method employed HAM1000 dataset, which included seven different types of cancerous lesions, including basal cell carcinoma, dermatofibroma malignancy, malignant melanocytic, benign melanomas, melanocytic lesions, and actinic keratosis, among others. Classification was carried out using a CNN model, which was 90.67% accurate [17]. In another study, machine learning and deep learning techniques for skin lesion classification and diagnosis were reviewed. It was concluded that although, machine learning techniques such as *k*-nearest neighbor (KNN), support vector machine (SVM), *k*-means clustering, and Naïve Bayes methods have been used for skin lesion classification, deep learning approaches such as CNN tend to outperform machine learning methods [18].

Researchers have also used image augmentation techniques for the identification of skin lesions, in particular, melanoma. A skin analysis system was proposed employing the synthetic minority oversampling technique (SMOTE) and used the deep CNN-based SqueezeNet model for classifying malignant skin melanoma, atypical nevus, and common nevus from a publicly available dataset, PH^2^. The results of the study exhibited an accuracy of 92.18% [19]. In another system, a psoriasis assessment system was proposed using algorithms including KNN, random forest (RF), deep neural network (DNN), Naïve Bayes, and SVM. A total of 80 psoriasis patch images were used, and the results demonstrated the highest accuracies of 98.6% and 92.6% achieved via RF and KNN, respectively [20]. In a similar study, Dash et al. [21] proposed a CNN model for the detection of psoriasis. A total of 5241 images of psoriasis lesions were used, and the findings of the study exhibited an accuracy of 94.80%. In another study, psoriasis skin image analysis was carried out with machine learning methods of KNN, SVM, RF, and CNN. A total of 90 images of psoriasis skin lesions were used, and the results demonstrated the highest accuracy of 95%, and 17% being achieved by CNN [22].

The literature review summarized in Table 1 shows that no work has been done for the identification of the five different types of psoriasis, including pustular, guttate, inverse, plaque, and erythrodermic. Previously, machine learning and deep learning algorithms have been used to analyze skin images from publicly accessible datasets. However, no work has been done using the Dermnet and Nanyang Technological University (NTU) databases that we employed in our proposed research to classify five kinds of psoriasis. Furthermore, no study on psoriasis categorization using both CNN and LSTM deep learning approaches has been done. As a result, using CNN and LSTM as deep learning techniques, we present an innovative application for classifying five distinct forms of psoriasis, including pustular, guttate, inverse, plaque, and erythrodermic.

## 3. Materials and Methods

### 3.1. Image-Based Datasets

#### 3.1.1. Normal Skin

A total of 172 images of different areas of body including hands, feet, back, chest, and legs have been collected from the NTU dataset. In particular, the Biometrics and Forensics Lab (BFL) NTU dataset was used. The BFL NTU dataset consists of skin images from different parts of the human body including hands, chest, back, inner forearm, inner thigh, and lower leg [23]. The BFL NTU dataset is a publicly available dataset with a normalization procedure applied so that the aspect ratio and size of each image are the same [23].  Figure 1 illustrates a sample image of normal skin used from the BFL NTU dataset.

#### 3.1.2. Psoriasis

A total of 301 images pertaining to five types of psoriasis have been obtained from the Dermnet dataset. The Dermnet dataset consists of 23 types of dermatological disorders, including plaque, guttate, inverse, pustular, and erythrodermic psoriasis. Other types of skin diseases comprise that of alopecia areata, poison ivy, and eczema [24].  Figure 1 represents few of the images of each of the five types of psoriasis that we used in this study.

*(1) Plaque psoriasis*. A total of 99 images of plaque psoriasis were retrieved from the Dermnet dataset [24]. Plaque psoriasis tends to appear on the skin surface in the form of thick and red patches [25].  Figure 1 represents a sample input image of plaque psoriasis used in this study.

*(2) Guttate Psoriasis*. A total of 96 gutatte psoriasis images were collected from the Dermnet dataset and used in this study. Guttate psoriasis is a form of skin infection that appears on the skin surface in tear-drop shaped red and itchy patches [26].  Figure 1 represents a sample input image of guttate psoriasis used in this study.

*(3) Inverse Psoriasis*. Inverse psoriasis also referred to as hidden psoriasis is a form of psoriasis that tends to infect the skin folds, areas where one skin region rubs against another skin region [27]. In this study, we used a total of 25 images of inverse psoriasis retrieved from the Dermnet dataset.  Figure 1 represents a sample input image of inverse psoriasis used in this study.

*(4) Pustular Psoriasis*. A total of 48 images of pustular psoriasis were used from the Dermnet dataset. White bumps filled with pus within or around red scaly patches are representative of pustular psoriasis [28].  Figure 1 represents a sample input image pustular psoriasis used in this study.

*(5) Erythrodermic Psoriasis*. A total of 33 images of erythrodermic psoriasis were retrieved from the Dermnet dataset and used in this study. Being one of severe types of psoriasis, erythrodermic psoriasis involves inflammation with peeling rashes that burn considerably [29].  Figure 1 represents a sample input image of erythrodermic psoriasis used in this study.

### 3.2. Proposed Deep Learning Technique with CNN and LSTM

The Pandas Python Library used in this study comprises of the Dataframe function that aids in organizing the sample input images and eliminates unwanted rows and columns. The code has been written with Python using a Linux workstation involving the use of the TensorFlow package. Two deep learning approaches, convolutional neural network (CNN) and long short-term memory (LSTM), are used to produce the classification methodology.  Figure 2 depicts the flow process of the proposed deep learning approach. It begins with normal skin and the five kinds of psoriasis, including plaque, inverse, guttate, pustular, and erythrodermic psoriasis, as input example images. Following that, an image enhancement procedure is used to remove distortion from the sample images. After the images are enhanced, they undergo segmentation after which the images are divided in training and testing samples. Empirical studies have demonstrated that more accurate and robust results can be acquired via 20% to 30% of the data being used for testing and 70% to 80% for training [30]. As a result, 80% of the input sample images are used to train the classification model, while the remaining 20% are used for validation and testing. The categorization of an image into guttate psoriasis (class 0), inverse psoriasis (class 1), erythrodermic psoriasis (class 2), normal skin (class 3), plaque psoriasis (class 4), and pustular psoriasis (class 5) represents the outcome of the proposed deep learning approach.

### 3.3. Preprocessing of Image

#### 3.3.1. Cleaning and Preparation of Dataset

Images retrieved from the BFL NTU and Dermnet datasets were cleaned by opening each image in order to identify that if it is clearly exhibiting the particular diseased part or not and then select the most authenticated images.

#### 3.3.2. Data Augmentation

In this study, data augmentation was executed by rotating each image to 15°, shifting height and width and horizontally flipping the image. We restricted our data augmentation up to some range, in particular 200 to 400 images, so that we could get similar number of images in each class. Data augmentation was done in order to overcome biasness issues; hence, we increased the size of our data and applied deep learning techniques on it.  Figure 3 exhibits the number of images for each class following data augmentation.

#### 3.3.3. Image Enhancement and Image Segmentation

Image enhancement is a technique involving improvement of the input images with overall enhancement of contrast, brightness, and pixel luminance values [31]. The sklearn.preprocessing package, which is part of scikit-image processing, contains a number of image enhancing algorithms. To improve the sample input images in this research, the image enhancement method of histogram equalization was used. Histogram equalization (HE) improves low-contrast sections of an image, resulting in images with increased overall contrast [32]. The HE approach is used in this work to transform RGB images into equivalent hue-saturation-value (HSV) image format. In addition, image segmentation was carried out using the edge detection approach. The edge detection technique involves identifying edges within an image and following change in the intensity values, and hence, this results in a segmented image [33]. The resize function is used in this study to resize input sample images to a 64 × 64 resolution. Moreover, the antialiasing technique included in Python's scikit-image processing package is also employed. In particular, the multisample antialiasing (MSAA) technique is used being denoted as true so that the rough edges in the input images are smoothened.

### 3.4. Splitting Dataset

Following image preprocessing, the data are separated into three portions in an 8 : 1 : 1 ratio, training, validation, and testing. Within this percentage, 80% of the images are used to train classification models, with the remaining 10% used for validation and testing. As shown in Table 2, 1468 training images of all five classes of psoriasis are used while 182 images are used for validation and 188 images are used for testing the classification models.

### 3.5. VGG-19 Pretrained CNN Model

A large network visual geometry group (VGG-19) pretrained CNN model consisting of 19 neural layers is used in this study. The VGG-19 is a deep CNN model used to classify images, and the arrangement of the layers are shown in Figure 4 [34]. The purpose of max-pooling is to down sample the expression of the inputs in order to minimize their computational sizes. Hence, max-pooling is responsible for decreasing the volume size. A pretrained CNN model was used in this study as for image classification, pretrained CNN models are available, and there was no need for training the model from scratch.

#### 3.5.1. Architecture of VGG-19 Pretrained CNN Model

Figure 4 exhibits the architecture of VGG-19 pretrained CNN model. The model represents that training is done layer by layer in which, convolutional layers with different filter sizes are present with some pooling layers which are responsible for reducing the volume for each next layer. Following the combination of pooling and convolution layers, a fully connected (FC) layer is formed with 4096 units along with a softmax output layer. Moreover, in this study, the VGG-19 pretrained CNN model is incorporated with some trainable layers in order to make the model work more accurately and efficiently. There are four convolution layers in the classification model, and a max-pooling process is preceded by each convolution layer. Such four convolution layers are used to diagnose the five psoriasis types through the extraction of features from the input sample images.

### 3.6. LSTM Model

As compared to the pretrained CNN model used, an LSTM model was trained from scratch as only time series-based pretrained LSTM models are available, and we required an image classification model in this study. In model training of LSTM, we have used 3 × 64 input layers in order to train the model. The LSTM model comprises of internal systems called gates that control the information flow. Throughout training of the classification models, the gates can interpret what data are important [35]. These gates involve sigmoid triggers and tanh activation function as well. Both of these were used in this study, with sigmoid squishing around 0 and 1 values, whereas tanh squishes values between −1 and 1 [35]. Sigmoid is used for output layer calculation, while tanh is used for hidden layers because of marginally smaller scale as compared to sigmoid. Its derivative range is also slightly bigger than sigmoid which is ideal for steady gradients [35]. Other gates in LSTM we have used are as follows:

- Forget gate to decide which information should be thrown away
- Input gate to update the state of each cell
- Cell state is multiplied by the forget vector point-wise
- Output gate determines the next hidden state

### 3.7. Extraction of Features

Each input sample image is used to extract attributes, such as color, texture, and shape for our research. The cv2 and skimage Python libraries were used to extract color, texture, and shape data in this investigation.

#### 3.7.1. Color Feature

This study uses the NumPy array function to turn the images into a list of RGB color pixel values. In order to get the average of the three colors (red, green, and blue), the cv2 package is used. Initially, the blue color channel's mean value is determined, followed by the mean values for the green and red color channels. As part of Python's cv2 module, the NumPy array is able to hold RGB images in reverse order; hence, each value corresponds to a different color channel.

#### 3.7.2. Texture Feature

Python's skimage and cv2 libraries have been loaded into this research in order to take use of the image processing capabilities of scikit. Using local binary patterns (LBPs), texture descriptors have been used to compute the local representation of a texture feature. The LBP operator integrates statistical and structural models of texture analysis, which have been traditionally considered distinct [36]. Microprimitives and associated statistical placement criterions have been used to define texture. A supplementary measure of local image contrast may be used in conjunction with the primitives if desired. This contrast quantifies the strength of the primitives [36]. Each pixel in the image is compared to the surrounding pixels in order to build the local representation that finally extracts the texture feature. The threshold values are multiplied by the weights assigned to the relevant pixels, and the total is calculated to generate an LBP code for the neighborhood pixels.  Figure 5 demonstrates how the contrast measure is generated from the input images. Averaging the grey levels below and above the central pixel is done by subtracting the average values. Two-dimensional LBP and contrast distributions are most suitable for the texture feature extraction of images.

#### 3.7.3. Shape Feature

These images were used to extract shape information using the Hu moment shape descriptor. A Python package called OpenCV has been used to import the Hu moment shape descriptor. The Hu moment shape descriptor is represented by equations (1) and (2), where *S* denotes the calculated Hu moment and *δ* represents the normalized central moment. The central moment is taken into account while calculating Hu moments because it assists in the movement of the image's center region towards the centroid area. Images may be analyzed using Hu moments, which measure the contour of the sample input image, and this results in a NumPy array of the images. In addition, the flatten function aids in the creation of the form feature vector by flattening the NumPy array.

(1) $$\begin{array}{c} S=\delta o+\delta 1, \end{array}$$

(2) $$\begin{array}{c} S={\left(\delta o-\delta 1\right)}^{2}+4\delta^{2}. \end{array}$$

### 3.8. Mathematical Operations of CNN and LSTM

Table 3 elaborates the mathematical operations of CNN and LSTM.

### 3.9. SPSS Analysis

IBM SPSS Statistics for Windows, Version 22.0 of the Statistical Package for Social Sciences (SPSS). Both CNN and LSTM accuracies produced by IBM Corp. were tested using the paired sampled *T*-test at Armonk, NY. Both CNN and LSTM had a total of 30 accuracy samples.

## 4. Results and Analysis

### 4.1. Evaluation of CNN Model

Figure 6 demonstrates the training and validation of the CNN model, and it can be concluded that model accuracy at the time of training was higher at each epoch, whereas during validation, it decreases, and at some intervals, the model accuracy goes quite low. The values of the model accuracy per epoch ranges in between 95% and 100% at the time of training, while at the time of validation, the value lies in between 65% and 80%.

Figure 7 exhibits CNN model loss versus epoch. This model loss exhibits how well the model is doing in each epoch. It can be observed that as the epoch increases, the validation loss increases while the training loss is quite low. By observing both the graphs simultaneously, it can be observed that when the model accuracy was decreasing the model loss was high, whereas when the model accuracy was increasing, model loss was decreasing. Hence, this demonstrates that model accuracy and model loss are inversely related as represented in equation (3).

The training of the CNN model was stopped at 100 epochs for model accuracy and 35 epochs for model loss. The reason to stop training at these values of epochs was the same computation of model accuracy and model loss values. This means that at 100 epochs and beyond, the same model accuracy value was being computed. Similarly, at 35 epochs and beyond, the same value of model loss was being generated. Furthermore, drop-out layer regularization was used for avoiding over-fitting and fine tuning the CNN model. Also, in order to measure the loss in the CNN model, the binary cross-entropy loss function was used.

(3) $$\begin{array}{c} \text{model accuray of CNN}\propto \frac{1}{\text{model loss of CNN}}. \end{array}$$

### 4.2. Model Evaluation of LSTM

Figure 8 demonstrates the training and validation of the LSTM model, and it can be concluded that model accuracy at the time of training was higher at each epoch as compared to validation. The graph also shows a rise in training and validation, as can be seen. Up to the 40th epoch, the model accuracy values for training and validation are almost identical, but after that, training gains an advantage over validation in terms of accuracy. The graph ranges are in between 20% and 100% for training and 20% and 70% for validation.

Figure 9 represents LSTM model loss and epoch. In both training and validation, it can be observed that model loss is decreasing which also reflects that model accuracy, and model loss have an inverse relationship as expressed by equation (4).

LSTM model training was stopped at 100 epochs for model accuracy and 35 epochs for model loss. The reason to stop training at these values of epochs was the same computation of model accuracy and model loss values. This means that at 100 epochs and beyond, the same model accuracy value was being generated. Similarly, at 35 epochs and beyond, the same value of model loss was being generated. Furthermore, drop-out layer regularization was used for avoiding over-fitting and fine tuning the LSTM model. Also, in order to measure the loss in the LSTM model, the binary cross-entropy loss function was used.

(4) $$\begin{array}{c} \text{Model accuray of LSTM}\propto \frac{1}{\text{Model loss of LSTM}}. \end{array}$$

### 4.3. Performance Evaluation

In the evaluation of CNN and LSTM, confusion matrices have been employed. Confusion matrix shown in Figure 10 shows the expected results for each of the six groups. A total of six classifications of psoriasis have been indicated by the numbers 0, 1, 2, 3, 4, and 5, which are guttate, inverse, erythrodermic, normal, plaque, and pustular. True positive is when the classifier correctly predicts the positive class, whereas true negative (TN) indicates correct prediction of the negative class by the classifier. False positive (FP) is when the classifiers incorrectly predict the positive class while false negative (FN) represents incorrect prediction of the negative class.

All six classes were evaluated on 188 different images that were created by the CNN algorithm and shown in Figure 11. Of the 188 images analyzed, 158 were correctly categorized, according to the study. This yielded an accuracy of 84.04%. Thirty-four images were classified as guttate psoriasis, 23 as inverse, 23 as erythrodermic, 28 as normal skin, 28 as plaque, and 22 images were classified as pustular psoriasis.

Figure 12 illustrates the LSTM-created confusion matrix, which reveals that 136 of the 188 images were correctly identified. This yielded an accuracy of 72.34%. Thirty images were classified as guttate psoriasis, 20 as inverse psoriasis, 19 as erythrodermic, and 26 images as normal skin, 25 as plaque, and 16 images were classified as pustular psoriasis.

Table 4 shows CNN and LSTM's performance and classification results.

The graphical illustration of accuracy outcomes of both the CNN and LSTM models are exhibited in Figure 13.

The results generated by SPSS analysis are demonstrated by equation (5) where 29 denotes the degrees of freedom, 20.216 is the *t* statistic value, and probability value (*p* value) is less than 0.001, indicating that there is a significant difference between the accuracies obtained via CNN and LSTM.

(5) $$\begin{array}{c} t\left(29\right)=20.216,p<0.001. \end{array}$$

### 4.4. Performance Metrics

TP, FP, TN, and FN are computed with the help of the sklearn library of Python [39]. Classification methods involve classification metrics namely, sensitivity, specificity, and accuracy, that aid in assessing the performance of deep learning algorithms. Sensitivity is the classification metric that permits evaluation of a model's ability to classify true positives of each available class. In order to measure sensitivity, it is necessary to divide the total of true positives and false negatives by the number of true positives [40]. An algorithm's actual negative rate, or specificity, helps to identify all of the negative classes that were correctly categorized by the algorithm, as well. The ratio of true negatives to the total of true negatives and false positives may be described as specificity [40]. It is possible to determine the accuracy metric by dividing the number of correctly categorized predictions by the total number of predictions [41]. In this study, the accuracy, sensitivity, and specificity metrics indicated by equations (6)–(8) were used to assess the performance of the CNN and LSTM models.  Table 5 shows the values of these performance indicators, determined according to their formulae.

(6) $$\begin{array}{c} \text{accuracy}=\frac{\text{TP}+\text{TN}}{\text{TP}+\text{FP}+\text{TN}+\text{FN}}*100\%, \end{array}$$

(7) $$\begin{array}{c} \text{sensitivity}=\frac{\text{TP}}{\text{TP}+\text{FN}}*100\%, \end{array}$$

(8) $$\begin{array}{c} \text{specificity}=\frac{\text{TN}}{\text{TN}+\text{FP}}\;*100\%. \end{array}$$

## 5. Discussion

### 5.1. Main Findings

The goal of this work was to extract characteristics such as color, texture, and form from databases of dermoscopic images of plaque, guttate, inverse, pustular, and erythrodermic psoriasis. The images were classified using deep learning methods such as convolutional neural networks (CNNs) and long short-term memories (LSTMs).

CNN works on pixel-by-pixel convolution, whereas LSTM runs on feedback mechanism. CNN learns each minute detail about each pixel value. On the contrary, LSTM is dependent on past inputs. The achieved accuracy of the CNN model as exhibited by Figure 13 is 84.2%, whereas LSTM accuracy is 72.3%. Figures 6 and 7 corresponding to the CNN model accuracy and model loss show that during training, CNN model accuracy was increasing and loss was near to 0%. Whereas in Figures 8 and 9, the LSTM model accuracy during training increases, while the loss decreases from 30% to 2%. CNN outperforms LSTM when it comes to categorizing skin images into the five categories of psoriasis and normal skin, according to our deep learning application.

Other techniques that have used similar deep learning methods have also achieved high accuracies. A skin lesion classification system was proposed using plaque psoriasis images with classification being executed by CNN, and the results of the study reported an accuracy of 60% [22]. Psoriasis was classified using dermoscopic images in another investigation. The study's findings showed that CNN had a precision rate of 92.9% [42]. Mathematical processing is the key to CNN's improved performance. Accordingly, the 84.2% accuracy achieved in this research using CNN is due to the usage of kernel convolution approach, which converts the data into higher dimensions and computes pixel-by-pixel transformation [43].

The specialty of our proposed deep learning application lies in being the first of its kind study encapsulating the classification of five different types of psoriasis and normal skin. A limitation of this study includes using publicly available datasets with no collection of clinical data. Hence, future work can be conducted using collected images from clinics and with other deep learning methods so that more robust classification performances can be accomplished.

## 6. Conclusion

In order to classify the five forms of psoriasis and normal skin, this research used a deep learning classification approach. Plaque, guttate, inverted, pustular, and erythrodermic are the five forms of psoriasis that may occur. Following the extraction of color, texture, and form characteristics, the convolutional neural network (CNN) and long short-term memory (LSTM) were used. The application of CNN presented an accuracy of 84.2% and that of LSTM presented an accuracy of 72.3%. The accuracies achieved demonstrate that the proposed deep learning application is reliable and effective. There are implications for further research in relation to the existing proposed deep learning application which can lead to enhancement of methods in biomedical imaging. The existing application can also be applied to other skin disorders along with being integrated with other deep learning techniques like RNN. Moreover, research pertaining to Psoriasis Area and Severity Index (PASI) scoring can also be carried out in the future.

## Figures and Tables

**Figure 1:** Images of normal skin and five kinds of psoriasis, including plaque, guttae, inverse, pustular, and erythrodermic, are shown in the examples.

**Figure 2:** Flow process of the proposed classification technique.

**Figure 3:** Dataset following data augmentation.

**Figure 4:** Architecture of the VGG-19 pretrained CNN model.

**Figure 5:** Contrast and LBP calculation.

**Figure 6:** CNN epoch versus model accuracy.

**Figure 7:** CNN epoch versus model loss.

**Figure 8:** LSTM epoch versus model accuracy.

**Figure 9:** LSTM epochs versus model loss.

**Figure 10:** Confusion matrix.

**Figure 11:** All six classes of CNN images are shown in a confusion matrix.

**Figure 12:** All six classes of LSTM images are shown in a confusion matrix.

**Figure 13:** Accuracies of CNN and LSTM.

**Table 1:** An overview of previously published cutting-edge research.

Year	Method	Skin disorder	Accuracy
2021	CNN [16]	Melanoma	97.16%
2021	RCNN [14]	Melanoma	96.3% (ISBI2016), 94.8% (ISBI2017), 88.5% (HAM1000)
2021	CNN [17]	Dermatofibroma, benign keratosis, basal cell carcinoma, melanoma, melanocytic nevi, actinic keratosis, and vascular	90.67%
2021	CNN [19]	Melanoma	92.18%
2021	RF and KNN [20]	Psoriasis	98.6% (RF) and 92.6% (KNN)
2019	CNN [21]	Psoriasis	94.80%
2018	CNN [15]	Melanoma	82.4%
2018	CNN [22]	Psoriasis	95.17%

**Table 2:** Number of training, testing, and validation images.

Serial number	Classes	Training images	Validation images	Testing images
1.	Normal skin	220	27	29
2.	Plaque psoriasis	316	39	40
3.	Inverse psoriasis	178	22	23
4.	Guttate psoriasis	306	38	39
5.	Pustular psoriasis	240	30	30
6.	Erythrodermic psoriasis	208	26	27
	Total	1468	182	188

**Table 3:** Mathematical operations of CNN and LSTM.

CNN	LSTM
CNNs are feed-forward neural networks in which learning is achieved pixel by pixel [37]. CNN employs convolution kernel *h*, a matrix that moves over the input images and executes a dot product with the central region of the input data, represented by *f∗h*. Following this, the output is yielded as matrix of the dot products with *m* columns and *n* rows and is represented by the following expression; $G\;\left(m,n\right)=\;f\;*\;h\;\left(m,n\right)=\sum_{j}\sum_{k}h\left[j,k\right]f\left(m-j,n-k\right).$	The LSTM deep learning algorithm involves working on a loop network that has two hidden states: cell state and hidden state. Furthermore, it involves assigning weights *W* as learning parameters for the classification algorithm [38]. *X*_2_ denotes the LSTM layers with the hidden layers being responsible for carrying feedback. The following expression exhibits how the algorithm works with sigmoid function *σ* and the inclusion of past values; $\begin{array}{c} \mathrm{Initial}\;\mathrm{Gate}=\sigma \;\left(W_{\mathrm{Input}}^{1}*X_{2}+W_{\mathrm{Past}}^{1}*\mathrm{Hidden}\;\mathrm{layer}\right),\\ \mathrm{Input}\;\mathrm{Gate}=\sigma \;\left(W_{\mathrm{Input}}^{2}*X_{2}+W_{\mathrm{Past}}^{2}*\mathrm{Hidden}\;\mathrm{layer}\right). \end{array}$
	Output Gate=*σ* (*W*_Input_^3^*∗X*_2_+*W*_Past_^3^*∗*Hidden layer).

**Table 4:** Classification results of CNN and LSTM.

Classes	CNN		LSTM	
	Test images	Truly classified	Test images	Truly classified
Normal skin	29	28	29	26
Plaque	40	28	40	25
Inverse	23	23	23	20
Pustular	30	22	30	16
Erythrodermic	27	23	27	19
Guttate	39	34	39	30
Total	188	158	188	136

**Table 5:** Values of performance metrics including sensitivity, specificity, and accuracy for all six classes.

Algorithm	Class	Sensitivity (%)	Specificity (%)	Accuracy (%)
CNN	0	82.0	71.0	84.2
CNN	1	100.0	95.0	84.2
CNN	2	85.0	85.0	84.2
CNN	3	96.0	100.0	84.2
CNN	4	70.0	90.0	84.2
CNN	5	73.0	75.0	84.2
LSTM	0	74.0	65.0	72.3
LSTM	1	86.0	83.0	72.3
LSTM	2	70.0	79.0	72.3
LSTM	3	89.0	100.0	72.3
LSTM	4	62.0	69.0	72.3
LSTM	5	53.0	55.0	72.3

## Data Availability

Data is available on request from the corresponding author.
